# High Expression of *SMO* and *GLI1* Genes with Poor Prognosis in Malignant Mesothelioma

**DOI:** 10.1155/2023/6575194

**Published:** 2023-04-24

**Authors:** Guan-Ying Ma, Shuai Shi, Yin-Zhou Sang, Ping Wang, Zhi-Gang Zhang

**Affiliations:** ^1^Department of Clinical Pathology, Chengde Medical University, Chengde, Hebei 067000, China; ^2^Department of Pathology, Cangzhou People's Hospital, Cangzhou, Hebei 061000, China

## Abstract

**Background:**

To investigate the value of *SMO* and *GLI1* genes in the hedgehog pathway in malignant mesothelioma specimens. Further study on the expression and prognosis of *SMO* and *GLI1* in malignant mesothelioma tissues and the relationship between the two and the molecular mechanisms of mesothelioma immunity and to further investigate the prognostic value of mesothelioma expression.

**Materials and Methods:**

Immunohistochemistry and RT-qPCR were applied to detect the expression of *SMO* and *GLI1* proteins and mRNA in biopsy specimens and plasma cavity effusion specimens from malignant mesothelioma (*n* = 130) and benign mesothelial tissues (*n* = 50) and to analyze the clinicopathological significance and survival risk factors of *SMO* and *GLI1* protein expression in mesothelioma. The mechanisms of mesothelioma cell expression and immune cell infiltration were investigated using bioinformatics methods.

**Results:**

*SMO* and *GLI1* in mesothelioma tissues detected high concordance between the diagnostic results of mesothelioma biopsy specimens and plasma cavity effusion specimens. The expression levels of *SMO* and *GLI1* protein and mRNA in mesothelioma tissues were higher than those in benign mesothelioma tissues. The expression levels of *SMO* and *GLI1* protein were correlated with the age, site, and asbestos exposure history of patients with mesothelioma. The expression levels of *SMO* and *GLI1* protein were correlated with the expressions of ki67 and p53 (*P* < 0.05). *SMO* and *GLI1* gene expression levels were negatively correlated with good prognosis in mesothelioma patients (*P* < 0.05). Cox proportional risk model indicated that protein expressions of invasion, lymph node metastasis, distant metastasis, staging, and genes were independent prognostic factors of mesothelioma. The GEPIA database showed the overall survival rate and the disease-free survival rate of mesothelioma patients in the high *SMO* and *GLI1* expression groups; the UALCAN database analysis showed lower *SMO* expression levels in mesothelioma patients with more pronounced TP53 mutations (*P* = 0.001); *GLI1* gene expression levels were strongly correlated with lymph node metastasis in mesothelioma patients (*P* = 0.009). Timer database analysis showed that the mechanism of immune cell infiltration was closely related to *SMO* and *GLI1* expression. The degree of immune cell infiltration was strongly correlated with the prognosis of mesothelioma patients (*P* < 0.05).

**Conclusion:**

The expression levels of both *SMO* and *GLI1* proteins were higher than those of normal mesothelial tissues, and the mRNA expression levels also changed in the same direction. *SMO* and *GLI1* gene expressions in mesothelioma were negatively correlated with age, site of occurrence, and history of asbestos exposure. Positive expression of *SMO* and *GLI1* was negatively correlated with patient survival. The Cox proportional risk model showed that gender, history of asbestos exposure, site of occurrence, *SMO*, and *GLI1* were independent prognostic factors for mesothelioma. The mechanism of immune cell infiltration in mesothelioma is closely related to the gene expression of both and the survival prognosis of mesothelioma patients.

## 1. Introduction

Malignant mesothelioma is a highly aggressive serous cavity malignancy. It is mainly seen in patients over 60 years of age and is more common in men [1, 2]. Mesothelioma occurs mainly in the pleura, accounting for more than 85% of cases, and peritoneal mesothelioma accounts for 10%. Most malignant mesotheliomas are associated with exposure to asbestos [3–5]. By and large, tumors begin as multiple small plasma membrane nodules, which then fuse with each other, leading to the fusion of the visceral and mural plasma membranes with each other and encapsulating the tumor site. Mesothelioma is divided into epithelioid, sarcomatoid, and biphasic components, with the epithelioid being the most common. The prevalence of malignant mesothelioma is increasing year by year, and the prognosis of mesothelioma patients is extremely poor, with only about 10% of mesothelioma patients surviving longer than 3 years and a median survival time of only about 13 months [6–8]. Because of the insidious clinical presentation of mesothelioma, most patients are already at an advanced stage at the time of diagnosis. In clinical practice, despite treatment with anthracycline and cisplatin-based chemotherapeutic agents, the 5-year survival rate of patients is still less than 15% [9]. There are still no particularly clear findings on the pathogenesis of mesothelioma; therefore, it is essential to find more appropriate diagnostic markers, and improving the accuracy of mesothelioma screening and diagnosis in the early and middle stages is an important method used to improve the prognosis of patient survival. The current clinical application of biopsy specimens for the diagnosis of mesothelioma is more invasive to the patient. Plasma cavity fluid specimens have the advantage of being less harmful to the patient and easier to perform. Most patients with malignant mesothelioma will have chest and ascites as clinical manifestations, and extraction of plasma cavity fluid will also reduce the impact of adverse clinical symptoms on the patient. The production of plasma cavity fluid specimens as cytology sections may have disadvantages in diagnosis such as too few cells, superimposed cell blocks, and easy desquamation. We have modified centrifuged plasma cavity effusions for early to midstage mesothelioma screening to provide some basis for improving the diagnostic sensitivity and survival prognosis of mesothelioma patients.

The hedgehog (Hh) signaling pathway is one of the important signaling pathways in vivo that regulate organ growth and development and controls tissues in vivo during embryonic development, maintaining their normal structure and function [10] The Shh signaling pathway is a key component of the Hh signaling family, one of the most widely studied Shh signaling pathways, consisting of Shh, *SMO* genes belonging to class F G protein-coupled receptors, and *GLI1* is a direct transcriptional activator downstream of the Hh signaling pathway. The binding of Hh ligands to the transmembrane receptor fragmentation protein-1 (PTCH-1), which has an inhibitory effect on *SMO* release, causes upregulation of activated *SMO* downstream of the GLI zinc finger to activate the Hh pathway and promotes fibroblast migration, invasion, and skin wound healing. According to Kaushal Jyoti et al. and Nastase et al.'s research, siRNA transfection tests showed that SMO promotes cell migration by acting upstream of the PI3K pathway [11, 12]. SMO operates upstream of phosphatidylinositol 3 kinase (PI3K)-c-Jun terminal kinase (JNK)-catenin to increase cell motility, according to western blot and siRNA transfection study. The fact that -catenin regulates Hh pathway genes including *SMO* and *GLI1* suggests that -catenin activates Hh signaling in turn [13, 14]. Through its new roles in controlling E-cadherin/-catenin regulation of cancer cell characteristics through the overexpression of the adhesive-forming protein MUC5AC, which interferes with the membrane location of E-cadherin, *GLI1* increases the motility and invasiveness of pancreatic ductal adenocarcinoma cells [15, 16]. Some graduate students have proposed a link between the Hh signaling system and mesothelioma based on evidence that the pathway is critical in the development of a number of malignancies; however, the results are conflicting. In this study, we examine the levels of protein and mRNA expression, survival prognosis, and immune cell infiltration mechanisms of important Hh pathway genes in malignant mesothelioma. These findings are important for the development and clinical treatment of malignant mesothelioma and offer new ideas for new gene therapy targets for malignant mesothelioma.

## 2. Materials and Methods

### 2.1. Data on Clinical Specimens

Pathological specimens from all enrolled patients were collected to obtain information about the patients' general condition, personal hygiene habits, underlying diseases, and type of work. The Ethics Committee (K2021-108 is the number of the ethics approval document) gave its approval for the study. 130 individuals with plasma cavity illness were chosen after screening to receive treatment at Cangzhou People's Hospital between January 2017 and December 2021. The pathological diagnosis complied with the clinical diagnosis and treatment recommendations for malignant mesothelioma in terms of diagnostic criteria. The following were the criteria for inclusion: informed agreement was obtained from patients and their families, and patients were followed up; the age range was 18 to 80; the histology type was patients with a definite pathological diagnosis of thoracoabdominal mesothelioma (epithelial). The official pathology report identified 4 specimens as having mesothelioma following the discovery of D2-40, WT1, and other markers. The following were the exclusion requirements: patients without genetic disorders in their family history medical records; patients with insufficient pathology data and lost to follow-up; (iii) patients with specimens contaminated due to improper handling of specimens in the experiment (inadequate fixation of specimens, antibody cross binding, etc.).

### 2.2. Immunohistochemical Study Methods

Immunohistochemistry was used to identify the expression of *SMO* and *GLI1* proteins in paraffin tissues. Retrospective analysis of the recruited patients was performed utilizing a diagnostic test evaluation approach. Diagnostic tests were administered to patients who met the inclusion and exclusion requirements, and the test findings were documented. Cases were renumbered using a double-blind approach after those who did not match the inclusion criteria were removed from the research. Four senior pathologists performed pathophysiological diagnoses on each case as part of a new round of diagnostic tests. Then, using immunohistochemical staining for *SMO* and *GLI1*, all cases were evaluated. Sensitivity and specificity of the newly developed combination diagnostic approach were recorded to determine the effectiveness of the diagnostic tests.

Use no less than 60 ml of naturally settled serum cavity fluid over a period of 0.5 hours, according to the modified procedure for paraffin sectioning of plasma cavity fluid. Six centrifuge tubes containing the serum luminal fluid samples were spun three times at room temperature (15–25°C) (depending on the size of the centrifuged precipitated cells). The first cycle of centrifugation takes place at 694 × g for 5 minutes, after which the supernatant is spread out and discarded. A few drops of protein, glycerol, and 90% ethanol are added during the second round of centrifugation to revive the precipitate. The precipitate is once more centrifuged for 5 minutes at 694 × g. The second centrifugation and the third centrifugation are identical. After centrifugation, the supernatant was discarded, and the cell blocks were removed, fixed, dehydrated, embedded, and sectioned. Malignant mesothelioma tissue and benign mesothelial tissue samples were collected, neutral formalin was fixed for 12-24 hours, and wax blocks were prepared by dehydration and paraffin embedding. The tissue sections are adhered to the slides at a thickness of 5 *μ*m, dried overnight at 56-60°C, and removed to cool to room temperature. Antigenic thermorepair preconditioning (EDTA) reagents are used. Then, conventional tissue paraffin sectioning, dewaxing solution, gradient alcohol hydration dewaxing, a special dyeing tank filled with 200 ml of EDTA buffer with pH 8.0, and a boiling water bath were used to put in dewaxed and hydrated slices and boiled for 20 minutes, kept warm for 10 minutes, cooled to room temperature (15-25°C), and washed with water; 3% H_2_O_2_ incubated at room temperature (15-25°C) for 10 minutes, PBS solution soaked; remove the PBS solution, add antibody reagent dropwise on the tissue paraffin section, so that the reagent covers the edge of the tissue, incubate in a constant temperature incubator at 37°C for 60 min, remove the reagent on the tissue, immerse the PBS solution for 3 min, and repeat 3 times; remove PBS solution, add anti-mouse/rabbit IgG peroxidase polymer dropwise, incubate for 30 min at room temperature (15-25°C), remove reagent, PBS solution immersion; add DAB chromogenic solution dropwise and incubate for 10 min at room temperature (15-25°C); hematoxylin counterstained for 10 sec, dehydrated, transparent with xylene, and sealed.

### 2.3. Immunohistochemical Reagents and Interpretation Criteria

The monoclonal antibody *SMO* (ab124964) against rabbit was obtained from Abcam Inc. The dilution used for immunohistochemistry (paraffin-embedded sections) was 1 : 1000, and the positive control was gastric cancer tissue. *GLI1*, a rabbit polyclonal antibody (product code ab217326; dilution 1 : 100), was obtained from Abcam, and the positive control was intestinal cancer tissue. Both antibodies are localized to the cytoplasm. Positive staining is brownish in color. Based on the results of the staining depth assessment, both experts verified the results of any discrepancies, ensuring consistency of the final conclusions.

The expression results were graded and counted as follows: the percentages of positive tumor cells were 0 (≤5%), 1 (6%-25%), 2 (26%-50%), 3 (51%-75%), and 4 (>75%). The staining intensity was graded as 0 (no staining), 1(+), 2(++), or 3(++++). Immunohistochemical results were scored according to the percentage of positive tumor cells multiplied by the staining intensity. The final immunostaining score for each section was 0-12, with a score of 0-4 being a low expression, while a score of 5-12 was a high expression.

### 2.4. RT-qPCR Reagent Companies and Procedures

Total RNA was extracted from the cells with a Trizol kit, and the concentration of each group of RNA was measured with a nucleic acid protein assay (repeated three times to take the average), and the RNA was reverse transcribed to cDNA according to the hair transcription system and conditions in the following table, and the system was as follows (Table 1).

The primers were synthesized by TianyiBiotech with the following sequences (Table 2).

Using the above cDNA as a template, the PCR primer sequences were identical to the above RT-qPCR primer sequences. The RNA concentration and purity were detected by taking 2 *u*l of RNA with a UV spectrophotometer, and the OD260/280 values were between 1.8 and 2.0. After calculation, the concentration of our extracted RNA was between 0.38-0.96 mg/ml. And the reaction system was as follows (Table 3).

The data is processed after the program is completed (Table 4).

The target gene was amplified by a two-step method.

### 2.5. Bioinformatics Analysis

GEPIA (http://gepia.cancer-pku.cn/) (gene expression profile data dynamic analysis) was developed by Peking University and applied to integrate and analyze cancer expression profile data. This interactive web server contains 9,736 tumor samples and 8,587 normal samples of 33 malignant tumors from TCGA and GTEx databases with RNA sequencing expression data to analyze the correlation between candidate genes and the survival and prognosis of colon cancer patients through survival curves. The Kaplan-Meier method was used to analyze the relationship between *SMO* and *GLI1* genes and the prognosis of mesothelioma patients and to draw survival curves. UALCAN (http://ualcan.path.uab.edu) is an online website for analyzing and mining the TCGA database, built on PERL-CGI, javascript, and CSS. It can analyze whether a gene is associated with cancer and paracancer, pathological grade, prognosis, and other factors in TCGA database samples. In this study, we used UALCAN software to analyze the malignant mesothelioma and benign mesothelial tissue data in the TCGA database. The relationship between immune cells and mesothelioma survival prognosis, mesothelioma with associated immune cell infiltration, and *SMO* and *GLI1* gene expression was based on the Timer database online website (http://http://timer.cistrome.org/).

### 2.6. Statistical Analysis

Statistical analysis was performed using SPSS 23.0 (IBM) statistical software. The correlation between SMO and GLI1 protein expression levels and mesothelioma clinicopathology was measured by correlation analysis, and the correlation between *SMO* and *GLI1* protein expression and mesothelioma clinicopathological characteristics was statistically significant by correlation 2/Fisher's test (*P* < 0.05). Correlation tests were performed using Spearman's rank correlation analysis; survival curves were plotted using GrapHD software. Multifactorial survival risk models established by Cox proportional regression risk analysis were statistically significant (*P* < 0.05).

## 3. Result

### 3.1. Expression and Correlation Analysis in Mesothelioma

HE sections of malignant mesothelioma show an epithelioid cell morphology, mostly round, rectangular, or polygonal, with abundant eosinophilic cytoplasm and mild nuclei (Figures 1(a)–1(d)). Statistical analysis of immunohistochemistry showed that *SMO* and *GLI1* were expressed in the cytoplasm. Statistical analysis showed that the positive expression of *SMO* in benign mesothelial tissue and malignant mesothelioma was 14.00% (7/50) and 81.54% (106/130) of biopsy specimens, respectively, with statistically significant differences (*P* < 0.05, Table 5); *GLI1* positivity was 18.00% (9/50) and 76.15% (99/130), respectively. The differences were statistically significant (*P* < 0.05, Table 5). According to the scoring criteria, the protein expression level was higher in malignant mesothelioma biopsy specimens than in benign mesothelial tissue, and the difference was statistically significant (*P* < 0.05) (Figures 1(e)–1(h)). In plasma cavity effusion specimens, *SMO* positive expression rates were 22.00% (11/50) and 73.08% (95/130) in benign mesothelial tissue and malignant mesothelioma, respectively (*P* < 0.05, Table 6); *GLI1* positive rates were 32.00% (16/50) and 66.15% (86/130), respectively, with statistically significant differences (*P* < 0.05, Table 6). *SMO* and *GLI1* protein expression levels were higher in mesothelioma plasma cavity effusion specimens than in benign mesothelial tissues (Figures 1(i)–1(l)).

After comparing the diagnosis of malignant mesothelioma in plasma cavity fluid specimens with that of biopsy specimens, we found a high level of agreement, and a comprehensive analysis of this new diagnostic method has a high clinical application. The results of Spearman's correlation analysis in 130 patients with malignant mesothelioma showed a positive correlation between *SMO* protein and *GLI1* protein expression in mesothelioma (*R* = 0.673) with statistically significant differences (*P* = 0.000, Table 7). Combining the above results showed a positive correlation between *SMO* expression and *GLI1* expression in mesothelioma tissues, which was statistically significant (*P* < 0.05). It is suggested that *SMO* may have a role in the production of *GLI1*.

### 3.2. Analysis of mRNA Expression of *SMO GLI1* in Malignant Mesothelioma

The amplification curve is a curve describing the dynamic process of RT-qPCR, which is normally S-shaped. During the course of the PCR experiment, the fluorescence signal intensifies as the target gene continues to amplify. The fluorescence amplification curve is divided into three phases, and only during the exponential amplification phase of the fluorescence signal, a logarithmic relationship exists between the logarithmic value of the PCR product volume and the starting template volume, allowing for quantitative analysis. The Ct value indicates the number of cycles in each reaction well when the fluorescence signal reaches a set threshold. It has been confirmed that the higher the starting copy number of the template, the smaller the Ct value, demonstrating that there is also a linear relationship between the logarithm of the starting copy number of the template and the Ct value of this template. The mean Ct value was calculated for all samples tested by replicate wells and used to quantify the target genes contained in the samples.

In this experiment, △CtCa represents the relative value of the expression of the target gene in malignant mesothelioma tissues and the expression of the internal reference, △CtCa = Ct mesothelioma target gene Ct (*SMO* and *GLI1*) mesothelioma internal reference GAPDH, △CtN represents the relative value of the expression of the target gene in benign mesothelioma tissues and the expression of the internal reference, △CtN = Ct benign mesothelioma target gene (*SMO* and *GLI1*) benign. The expression of the target gene in malignant mesothelioma tissues was higher than that in benign mesothelioma tissues if △CtCa < △CtN, and lower than that in benign mesothelioma tissues if △CtCa > △CtN. After statistical analysis, △CtCa and △CtN both conformed to normal distribution. △CtCa < △CtN indicated that the expression of *SMO* and *GLI1* in mesothelioma tissues was higher than that in benign mesothelioma tissues; △CtCa > △CtN indicated that the expression in mesothelioma tissues was lower than that in benign mesothelioma tissues, and *P* < 0.05 was statistically significant.

In this experiment, the expression of ploidy of mesothelioma tissues compared with benign mesothelial tissues was meaningful when it was greater than or equal to 2 fold and not meaningful when it was less than 2 fold. The relative expression of mesothelioma tissue compared to benign mesothelial tissue was expressed by △△Ct, i.e., △△Ct = △CtA − △CtB = (Ct mesothelioma target gene − Ct mesothelioma endogene XX) − (Ct benign mesothelioma target gene − Ct benign mesothelial tissue endogene XX). Using *X* to denote the expression fold of mesothelioma tissue compared to benign mesothelial tissue, then X = 2ΔΔCt, when X ≥ 2, ΔΔCt ≥ 1, indicating that the expression of target gene (*SMO* and *GLI1*) in malignant mesothelioma tissue is higher than that in benign mesothelial tissue; when X < 2, ΔΔCt < 1, indicating that the expression of target gene (*SMO*, *GLI1*) in malignant mesothelioma tissue is the expression in malignant mesothelioma tissues was lower than that in benign mesothelial tissues.

In this experiment, a total of 30 tissue specimens were collected, and the statistical results showed that *SMO* was highly expressed in 28 mesothelioma tissues, with upregulation of more than 2 fold in 24 of the highly expressed samples, no significance in 4 cases, and lower expression than benign mesothelioma tissues in 2 cases (Figures 2(a) and 2(b)); *GLI1* was highly expressed in 27 mesothelioma tissues, with upregulation of more than 2 fold in 22 of the highly expressed samples, no significance in 5 cases, and lower expression than benign mesothelioma tissues in 3 cases (Figures 2(c) and 2(d)). *GLI1* was highly expressed in 27 mesothelioma tissues and upregulated up to 2 fold or more in 22 of the highly expressed samples, 5 cases were not significant, and 3 cases had lower expression in mesothelioma tissues than benign mesothelial tissues (Figures 2(c) and 2(d)).

RT-qPCR was applied to detect *SMO* and *GLI1* mRNA levels in malignant mesothelioma tissues and normal mesothelial tissues, and statistical analysis showed that *SMO* and *GLI1* mRNA expression levels were significantly higher in mesothelioma tissues than in normal mesothelial tissues (*P* < 0.05).

### 3.3. Analysis of Clinicopathological Data and Survival Prognosis

Statistical analysis of *SMO* and *GLI1* protein expression and clinicopathological data showed that the expression levels in patients with malignant mesothelioma were negatively correlated with age, history of exposure to asbestos chemicals, mesothelioma site, Ki67, and P53 expression (*P* < 0.05) and not significantly correlated with patient gender (*P* > 0.05). High protein expression cases were mostly seen in middle-aged and elderly people (*P* < 0.05, Table 8).

130 patients with effective malignant mesothelioma were followed up with a survival period of 2 ~ 55 months. Survival curves were plotted, and the analysis of *SMO* and *GLI1* protein expression was negatively correlated with good patient prognosis, with statistically significant differences (*P* < 0.05, Figures 2(e) and 2(f)). In univariate analysis, patient gender and history of asbestos exposure were associated with patient prognosis (*P* < 0.05, Table 9). Cox analysis showed that *SMO* and *GLI1* gene expression levels, site of tumorigenesis, patient gender, and history of asbestos exposure were risk factors for survival time in mesothelioma patients (*P* < 0.05, Table 10).

### 3.4. Bioinformatics Analysis Results

GEPIA database analysis showed that the overall and disease-free survival rates of mesothelioma patients in the *SMO* and *GLI1* high expression groups were significantly lower than those in the low expression group, with statistically significant differences (*P* < 0.05, Figures 3(a)–3(d)). The more obvious the mutation, the lower the *SMO* expression level (*P* = 0.001, Figure 3(e)); *GLI1* gene expression level was closely related to lymph node metastasis in mesothelioma patients, especially in N1 and N3, and the higher the number of lymph node metastasis, the lower the *GLI1* gene expression level (*P* = 0.009, Figure 3(f)).

Timer database analysis revealed that immune cell infiltration mechanisms in malignant mesothelioma were closely associated with *SMO* and *GLI1* expression. Immune cells with a high degree of infiltration in malignant mesothelioma tissues included CD4+T memory dormancy cells, CD4+T memory activation cells, macrophage M0, macrophage M1, and macrophage M2. The degree of immune cell infiltration was strongly correlated with the prognosis of mesothelioma patients. We found that B cells, CD8+ T cells, CD4+ T cells, neutrophils, and dendritic cells among immune cells were negatively correlated with *SMO* gene expression. Macrophages were positively correlated with *SMO* (*P* < 0.05, Figure 4(a)). Among *GLI1* gene expression in malignant mesothelioma, B cells and macrophages were positively correlated with *GLI1* gene expression, and the remaining immune cells were negatively correlated with *GLI1* gene expression (*P* < 0.05, Figure 4(b)). Meanwhile, we found that immune cell infiltration was closely related to the prognosis of mesothelioma patients. The higher the degree of neutrophil infiltration, the longer the survival time of mesothelioma patients, which was positively correlated (*P* = 0.001, Figure 4(c)), and the rest of the cells were less correlated with the prognosis of mesothelioma patients. For comparison of gene and immune cell survival analysis, cancer patients were automatically divided into high-and low-expression groups based on expression values. *SMO* and protein expression of *GLI1* genes had a significant effect on the survival prognosis time of patients with mesothelioma. Higher SMO expression levels were associated with a shorter survival time and a poorer prognosis for patients with mesothelioma (*P* = 0.005, Figure 4(d)). Among the copy number variants in mesothelioma, diploid/normal immune cells (B cells, CD8+ T cells, neutrophils, and dendritic cells) was higher than arm-level deletion and arm-level increase (Figure 4(e)). Interestingly, the higher the level of *GLI1* expression, the shorter the survival time and the worse the prognosis of patients with mesothelioma (Figure 4(f)), respectively. Among the copy number variants in mesothelioma, diploid/normal was higher in immune cells (B cells, CD8+ T cells, neutrophils, and dendritic cells) than arm-level deletion and arm-level gain (Figure 4(g)).

## 4. Discussion

Malignant mesothelioma has few treatment options due to its dysfunctional mutant state, and only about 12% of patients with malignant mesothelioma survive longer than 3 years, and its development may be closely related to occupational or environmental asbestos exposure [17], which is consistent with the pathological characterization of our experimental cases. The hedgehog (Hh) signaling pathway is associated with DNA methylation, histone modification, and other chromatin remodeling events that are closely associated with many cellular processes, including differentiation, development, and tumorigenesis. Previous studies found that the Hh pathway genes, *SMO* and *GLI1*, are regulated by bFGF, and the *SMO* receptor is responsible for maintaining normal embryonic development and that abnormalities in this protein are associated with cancer. Upregulation of *SMO* activates the Hh pathway, which then triggers the transcription of target genes through the transcription factor *GLI1* Kruppel family [18]. bFGF and Shh stimulate bone marrow-derived endothelial progenitor cells to proliferate, migrate, and produce vascular endothelial growth factor (VEGF), thereby promoting neovascularization of ischemic tissues [19]. In addition, the Shh pathway mediates the production and activation of matrix metalloproteinase 2 through the adhesion kinase/AKT signaling pathway, inducing cell migration and invasion in hepatocellular carcinoma. *SMO* acts upstream of PI3K-JNK signaling, and *β*-catenin is involved in a feedback mechanism regulating Hh pathway gene transcription. It is a positive regulator of Hh pathway gene transcription [20, 21]. In the experiments of this paper, we also found that the expression levels of *SMO* and *GLI1* proteins were higher in malignant mesothelioma tissues than in benign mesothelioma tissues, and by Spearman's correlation analysis, we found that *SMO* and *GLI1* were positively correlated in mesothelioma, which is consistent with the above findings and provides some basis for the upstream and downstream relationship between *SMO* and *GLI1* genes in mesothelioma. In pancreatic cancer, *GLI1* regulates EMT through specific target genes such as TGF-*β*, Ras, Wnt, P13K/AKT, and S100A4. Mutation or abnormal expression of *SMO* or Hh genes can lead to cell-specific proliferation and involvement in tumorigenesis and development. Mutation or abnormal expression of *SMO* or *Hh* genes can lead to cell-specific proliferation, and involvement in tumor development, with basal cell carcinoma, lung cancer, or breast cancer, is closely related [22]. In this study, we showed that *SMO* and *GLI1* genes have a key role in tumor development, and our experimental results also showed that the *GLI1* gene and its upstream *SMO* gene have a greater prognostic impact on mesothelioma patients, and we found that the survival time of mesothelioma patients was significantly longer when *SMO* and *GLI1* genes were lowly expressed. While *SMO* and *GLI1* expression levels were associated with mesothelioma patients, Balancin et al., Shoji et al., and Maio et al. found that the occurrence and prognosis of malignant mesothelioma were associated with multiple factors, and risk factors for death were determined by multivariate Cox regression, and their study table showed that younger age, female, epithelioid histology, and multimodal treatment all improved patient survival [23–25]. Our experiment confirmed that the patient's gender and history of asbestos exposure were associated with the patient's prognosis (*P* < 0.05). *SMO* and *GLI1* gene expression levels, tumor site, patient's gender, and history of asbestos exposure were all risk factors for survival time in mesothelioma patients (*P* < 0.05), and the findings were consistent with greater significance for the prognostic value of mesothelioma. Hotta and Fujimoto and Keshava et al. showed that poor prognosis of malignant mesothelioma is usually associated with immune T-lymphocyte infiltration [26, 27], which often inactivates tumor suppressor genes (TSG), including purex deletion and inactivation of various genetic alterations, but there is a lack of effective treatment options for mesothelioma patients, and only conventional chemotherapy is available. Inaguma et al. and Popat et al. found that immune cell evasion mechanisms are closely associated with malignant mesothelioma, such as a tightly regulated interaction between CD70 and CD27, which exerts a costimulatory effect through the NF*κ*B pathway to promote the expansion and differentiation of T cells. Immune evasion of malignant cells is closely associated with high CD70 expression, and overall survival of patients with CD70-expressing tumor cells is significantly reduced [28, 29]. Tumor-infiltrating lymphocytes (TIL) are potential independent risk factors for MPM patients, and in vitro experiments and immunodeficient mouse models suggest that immune cells may play a role in the immune evasion mechanism of tumors [30, 31]. Our analysis also showed that immune cell infiltration mechanisms were associated with *SMO* and *GLI1* expression, and that CD4+ T cells, neutrophils, and macrophages have an important impact on mesothelioma development and prognosis. We also found that immune cells are closely associated with the copy number immune mechanism of mesothelioma, which contributes to the prognostic assessment and targeted therapy of mesothelioma.

At present, biopsy specimens are mostly used clinically to diagnose mesothelioma, because mesothelioma cells are indistinguishable from degenerated or proliferating mesothelioma cells, and most patients with malignant mesothelioma effusion in the thorax and abdomen are already in advanced stages at the time of diagnosis, and cytological sections have disadvantages such as superimposed cell obstruction, high false-positive rate, and easy desquamation. We have improved the method by separating the plasma cavity fluid from the pericardium in paraffin sections, and the resulting cells are flattened, the sections are clearly stained, and the diagnostic results are accurate and easy to distinguish, providing an important basis for an accurate cytologic diagnosis of malignant mesothelioma. At present, the definite diagnosis of mesothelioma is mostly obtained by tumor resection or puncture specimens, and pathological specimens are not easy to obtain and harmful to patients; specimens of pleural and peritoneal fluid are easy to obtain and less harmful to patients, and the extracts can alleviate patients' clinical symptoms, which has obvious superiority. In our experiments, we also compared the results of biopsy specimens and effusion specimens, and the accuracy of the two detection methods was consistent, so the use of plasma cavity fluid specimens for the diagnosis of mesothelioma is a relatively novel method. However, the diagnostic accuracy may be slightly lower because of the low cell content in plasma cavity fluid, poor heterogeneity of exfoliated cells, and possible differences in cells in the fluid at different times, in which the accuracy of the location of the extracted fluid may affect the diagnostic accuracy of plasma cavity fluid specimens, but plasma cavity fluid specimens are superior to puncture biopsy, noninvasive, easy to operate, easy to obtain for clinical sampling requirements, and less painful for patients. Moreover, the prevalence of malignant mesothelioma has increased year by year in recent years due to industrialization and environmental changes, with increasing exposure to asbestos chemicals as risk factors, so plasma cavity fluid specimens can be used as an important tool for screening patients with mesothelioma and are of great importance for the clinical diagnostic value of malignant mesothelioma. In summary, *SMO* and *GLI1* genes are differentially expressed in malignant mesothelioma and benign mesothelioma tissues, which have more important guiding significance for the diagnosis and prognostic mechanism of mesothelioma and also open up new ideas for gene targeting and personalized immunotherapy of mesothelioma.

## 5. Conclusion

In conclusion, this study analyzed the relationship between *SMO* and *GLI1* expression prognosis and immune cell infiltration mechanisms in malignant mesothelioma tissues by immunohistochemistry, RT-qPCR, and bioinformatics. *SMO* and *GLI1* genes were correlated with gender, age, tumor site, history of asbestos exposure, and staging of mesothelioma patients. Expression levels of both were associated with poor prognosis of mesothelioma and infiltration of immune cells such as CD4+T. This study evaluated the factors affecting the development of malignant mesothelioma, proposed a new idea of *SMO*, *GLI1*, and immune cells as possible indicators of personalized immunotherapy and prognosis, and provided an experimental basis for finding new gene targets for mesothelioma.

## Figures and Tables

**Figure 1:** HE staining results of malignant mesothelioma biopsy (a) and reactive mesothelioma biopsy (b) (×200). HE staining results of malignant mesothelioma plasma cavity fluid specimens (c) and benign mesothelial tissue plasma cavity fluid specimens (d) (×200). *SMO* expression in mesothelioma biopsy specimens (e) and benign mesothelial tissue biopsy specimens (f) (×200). High expression of *GLI1* in mesothelioma biopsy specimens (g) and low expression in benign mesothelial tissue (h) (×200). Expression of *SMO* antibodies in mesothelioma plasma membrane effusion specimens (i) and benign mesothelial tissue (j) (×200). *GLI1*-expressing antibody in plasma membrane cavity effusion specimens from mesothelioma (k) and benign mesothelial tissue (l) (×200).

**Figure 2:** *SMO* mRNA expression levels in 30 malignant mesothelioma tissues (a). Total ratio of *SMO* mRNA expression levels in malignant mesothelioma tissues (b). *GLI1* mRNA expression levels in 30 malignant mesothelioma tissues (c). Total ratio of *GLI1* mRNA expression levels in malignant mesothelioma tissues (d). Survival analysis of patients with *SMO* gene expression levels (*P* < 0.0001) (e). Survival analysis of patients with malignant mesothelioma with *GLI1* gene expression levels (*P* = 0.0021) (f). N: malignant mesothelioma; C: benign mesothelial tissue.

**Figure 3:** Relationship between *SMO* gene expression levels and overall survival (a) and disease-free survival (b) of patients with malignant mesothelioma in the GEPIA database. Relationship between *GLI1* gene expression levels and overall survival (c) and disease-free survival (d) of patients with malignant mesothelioma in the GEPIA database. The relationship between *SMO* expression levels and mesothelioma TP-53 mutation status in the UALCAN database (e). The relationship between *GLI1* expression and lymph node metastasis in malignant mesothelioma (f).

**Figure 4:** Correlation between *SMO* expression levels and immune cells (CD4+ T cells, macrophages, B cells, CD8+ T cells, neutrophils, and dendritic cells) in malignant mesothelioma (a). Correlation between the level of *GLI1* expression and 8 immune cells in malignant mesothelioma (b). Correlation between the level of immune cell infiltration and the survival prognosis of mesothelioma patients (c). Correlation between *SMO* gene expression and the survival prognosis of mesothelioma patients (d). This is the relationship between *SMO* copy number variation and immune cell infiltration in malignant mesothelioma (e). The degree of correlation between *GLI1* gene expression and survival prognosis of mesothelioma patients (f). This is the relationship between *GLI1* copy number variation and immune cell infiltration in malignant mesothelioma (g).

**Table 1:** Retrotranscriptional response system and reaction conditions.

The reverse transcription system	Reaction conditions	
5 × g DNA digester buffer (2 *u*l)	42°C	2 min
gDNA digester (1 *u*l)	42°C	2 min
Template RNA (1 *u*l)	42°C	2 min
RNase-free H_2_O (6 *u*l)	42°C	2 min
2XHifair II SuperMix plus (10 *u*l)	25°C	5 min
	42°C	30 min
	85°C	5 min

**Table 2:** Primer sequence.

*SMO*	F: 5′-CCCTTGGTTCGGACAGACA-3′
	R: 5′-AAAGAAGCACGCATTGACG-3′
*GLI1*	F: 5′-CCAACTCCACAGGCATACA-3′
	R: 5′-AGATTCAGGCTCACGCTTC-3′
GAPDH	F: 5′-TCTGATTTGGTCGTATTGGG-3′
	R: 5′-GGAAGATGGTGATGGGATT-3′

**Table 3:** Reaction system.

F	0.4 *u*l
R	0.4 *u*l
ddH_2_O	7.2 *u*l
SYBR	10 *u*l
Template DNA	2 *u*l

**Table 4:** Reaction procedures and conditions.

Cycle steps	Temperature	Time	Cycle number
Premutability	95°C	5 min	1
Transgender	95°C	10 sec	40
Annealing/extension	60°C	30 sec	
Dissolution curve	Instrument default settings		1

**Table 5:** Biopsy specimen pathological morphology combined with immunohistochemical staining of *SMO* and *GLI1* results.

Category	CDKN2A (FISH)		*χ* ^2^	*P*	*SMO*		*χ* ^2^	*P*	*GLI1*		*χ* ^2^	*P*
	Positive (%)	Negative (%)			Positive (%)	Negative (%)			Positive	Negative (%)		
Mesothelioma	86.92	13.08	98.871	≤0.001	81.54	18.46	70.491	≤0.001	76.15	23.85	50.885	≤0.001
Mesenchymal hyperplasia	8.00%	92.00%			14.00	86.00			18.00	82.00		

**Table 6:** Results from the diagnosis of serous effusion samples detected by immunohistochemical staining of *SMO* and *GLI1*.

Category	CDKN2A (FISH)		*χ* ^2^	*P*	*SMO*		*χ* ^2^	*P*	*GLI1*		*χ* ^2^	*P*
	Positive (%)	Negative (%)			Positive (%)	Negative (%)			Positive	Negative (%)		
Mesothelioma	85.38	14.62	73.786	≤0.001	73.08	26.92	38.913	≤0.001	66.15	33.85	17.154	≤0.001
Mesenchymal hyperplasia	18.00	82.00			22.00	78.00			32.00	68.00		

**Table 7:** Correlation results of expression of SMO and GLI1 in mesothelioma.

Gene	Expression	*GLI1*		*r*	*P*
		Positive	Negative		
SMO	Positive	99	7	0.673	≤0.001
	Negative	6	18		

**Table 8:** Relationship between expression of *SMO* and *GLI1*protein and clinicopathological.

Clinical features	*N*	*SMO*		*χ* ^2^	*P*	*GLI1*		*χ* ^2^	*P*
		Negative	Positive			Negative	Positive		
Gender		24	106			31	99		
Male	60	8	52	1.947	0.163	12	48	0.908	0.341
Female	70	16	54			19	51		
Age (years)									
<60	39	3	36	4.292	0.038	4	35	5.666	0.017
≥60	91	21	70			27	64		
Asbestos exposure history									
Yes	85	4	81	30.866	≤0.001	12	73	12.798	≤0.001
No	45	20	25			19	26		
Pathological changes									
Pleural	60	3	57	13.414	≤0.001	8	52	6.781	0.009
Peritoneal	70	21	49			23	47		
Ki67									
Negative	36	18	18	32.898	≤0.001	23	13	43.960	≤0.001
Positive	94	6	88			8	86		
P53									
Negative	51	18	33	15.796	≤0.001	19	32	8.309	0.004
Positive	79	6	73			12	67		

**Table 9:** Univariate analysis of prognostic risk factors for malignant mesothelioma.

Clinical features	*N* (%)	95% CI (*SMO*)	*P* (*SMO*)	95% CI (*GLI1*)	*P* (*GLI1*)
Sex					
Male	60	2.723 (1.149-6.454)	0.023	3.080 (1.311-7.235)	0.01
Female	70				
Age (years)					
<60	39	0.653 (0.274-1.554)	0.335	0.650 (0.272-1.552)	0.332
≥60	91				
Asbestos exposure history					
Yes	85	0.331 (0.128-0.857)	0.023	0.269 (0.099-0.732)	0.010
No	45				
Pathological changes					
Pleural	60	0.521 (0.204-1.328)	0.172	0.730 (0.325-1.643)	0.447
Peritoneal	70				
P53					
Negative	51	0.506 (0.222-1.151)	0.104	0.619 (0.277-1.386)	0.244
Positive	79				

**Table 10:** Clinicopathological multivariate analysis of survival in patients with malignant mesothelioma.

Clinical features	95% CI (SMO)	*P* (*SMO*)	95% CI (*GLI1*)	*P* (*GLI1*)
Gender				
Male	0.407 (0.164-1.008)	0.052	0.316 (0.127-0.786)	0.013
Female				
Age (years)				
<60	1.196 (0.478-2.990)	0.038	1.040 (0.412-2.623)	0.934
≥60				
Asbestos exposure history				
Yes	5.855 (1.225-27.989)	0.027	6.990 (1.656-29.512)	0.008
No				
Pathological changes				
Pleural	3.049 (1.062-8.757)	0.038	2.471 (0.939-6.503)	0.067
Peritoneal				
P53				
Negative	1.103 (0.323-3.769)	0.876	0.904 (0.286-2.862)	0.864
Positive				
*SMO*				
Negative	13.240 (3.294-53.219)	≤0.001	/	/
Positive				
*GLI1*				
Negative	/	/	10.090 (2.969-34.294)	≤0.001
Positive				

## Data Availability

The data sets generated and/or analyzed in the present study can be obtained from the data storage repository of Cangzhou People's Hospital (Cangzhou, China) upon reasonable request (K2021-108).
